# Population Pharmacokinetics of Enteric-Coated Mycophenolate Sodium in Children after Renal Transplantation and Initial Dosage Recommendation Based on Body Surface Area

**DOI:** 10.1155/2022/1881176

**Published:** 2022-09-10

**Authors:** Guangfei Wang, Qiaofeng Ye, Yidie Huang, Hong Xu, Zhiping Li

**Affiliations:** ^1^Department of Clinical Pharmacy, National Children's Medical Center, Children's Hospital of Fudan University, Shanghai 201102, China; ^2^Department of Nephrology, National Children's Medical Center, Children's Hospital of Fudan University, Shanghai 201102, China

## Abstract

**Objective:**

Enteric-coated mycophenolate sodium (EC-MPS) is widely used in renal transplant recipients. There is a lack of study on the pharmacokinetics of this drug in children. This study is aimed at developing a population pharmacokinetic model of mycophenolic acid in children who were treated with EC-MPS after renal transplantation and to recommend initial dosage.

**Methods:**

Pediatric patients who had undergone renal transplantation and received EC-MPS were included. Data on demographic characteristics, biochemical tests, blood routine examinations, mycophenolic acid plasma concentrations, dosing amount and frequency of EC-MPS, and coadministered medications were retrospective collected from June 2018 to August 2019. Nonlinear mixed effect modeling methods were adopted to develop a population pharmacokinetic model with the data above. Additional data from September 2019 to July 2020 were used to validate the model. Simulations under different dosage regimen were conducted to evaluate the percentage of target attainment (PTA, AUC_0-12h_ 30–60 mg·h/L).

**Results:**

A total of 96 pediatric patients aged at 13.3 (range 4.3–18.0) years were included in the modeling group. Data from 32 patients aged at 13.0 (range 3.6–18.3) years were used to validate the model. A one-compartment model with a double extravascular absorption was developed. Body surface area (BSA) was added as a covariate. Simulations showed that for different dosing regimens, the highest percentage of target attainment is around 50%. The best dosing regimen is 180 mg every 48 hours for patients with BSA of 0.22–0.46 m^2^, 180 mg every 24 hours with BSA of 0.47–0.67 m^2^, 180 mg every 24 hours with BSA of 0.68–0.96 m^2^, 360 mg every 24 hours with BSA of 0.97–1.18 m^2^, 540 mg every 24 hours with BSA of 1.19–1.58 m^2^, and 360 mg every 12 hours with BSA of 1.59–2.03 m^2^.

**Conclusion:**

BSA could affect the area under curve of mycophenolic acid with the administration of EC-MPS. Considering the inflexibility of the dosage form, future development of smaller amount per tablet suitable for younger children with BSA < 1.19 m^2^ is warranted.

## 1. Introduction

Since 1954, when Joseph Murray performed the world's first successful renal transplant on the adult identical twin brothers, renal transplantation has become a preferred therapy in adult patient with irreversible renal failure [1]. However, children were still allowed to die of renal failure 60 years ago, which was due to ethical considerations of the benefits versus risks [1]. While part of renal transplantation was similar between children and adults, there were great technical challenges in small children [1–3]. Many of initial transplants failed because of inappropriate immunosuppression [1]. Appropriate use of immunosuppressants is of vital importance in the treatment of renal transplant patients. Immunosuppressants that have been developed and applied include corticosteroids, azathioprine, cyclosporin, tacrolimus, and mycophenolate mofetil (MMF) [1, 4]. MMF was developed in 1994 and has almost replaced azathioprine universally over the past two decades [5].

MMF is a prodrug that undergoes rapid hydrolyzation to the active metabolite mycophenolic acid (MPA) following oral administration [6, 7]. The major MPA is further transformed to the 7-*O*-mycophenolic acid glucuronide (MPAG), which is inactive but exhibits enterohepatic recirculation (EHC) that can cause the double absorption pharmacokinetic (PK) process [8]. The minor part of MPA is later metabolized to acyl-glucuronide (AcMPAG) [9]. MPA selectively and reversibly inhibits an enzyme called inosine monophosphate dehydrogenase (IMPDH), which plays a key role in the de novo purine biosynthesis [7, 10]. By blocking the pathway above, MPA inhibits T and B lymphocytes from proliferating, thus causing immunosuppression to prevent graft rejection [7].

Gastrointestinal reactions are frequently observed adverse effects caused by MMF in patients who undergo kidney transplantation [8, 11]. To decrease the gastrointestinal adverse reactions, EC-MPS was introduced [8]. EC-MPS (720 mg twice daily) was comparable to MMF (1000 mg twice daily), with similar profiles of efficacy and safety proven in two clinical trials [12, 13]. Area under the MPA concentration-time curve from 0 to 12 hours (AUC_0-12h_) was often used to estimate the exposure to MPA, with the consensus target between 30 and 60 mg·h/L for renal transplant recipients [14–16]. Although the AUCs are similar between administration with EC-MPS (720 mg) and MMF (1000 mg), pharmacokinetic profiles of the two are quite different as previously reported [8, 17]. Compared to MMF, the predose plasma concentrations of MPA were reported to be higher and peak concentrations to be lower with the administration of EC-MPS [15, 17]. In addition, the absorption process has more interindividual variability with EC-MPS than with MMF therapy [8]. Therefore, EC-MPS and MMF are different not only chemically but also in their pharmacokinetic process.

A lot of studies have reported the PK characteristics of MMF in both adult and pediatric patients using population pharmacokinetic (PPK) modeling strategies [6, 18–22]. However, few PPK models of MPA have been developed for EC-MPS treatment [8], especially in the pediatric population. Although EC-MPS and MMF have the same active component MPA, the PPK model developed for MMF may not fit EC-MPS. In addition to the lack of PPK models for EC-MPS administration in children, the dosing recommendation could be more accurate based on a proper PPK model. In the “Pediatric & Neonatal Dosage Handbook,” the dosing recommendation based on body surface area (BSA) for children after renal transplantation is 400 mg/m^2^/dose twice daily for children ≥ 5 years old [23]. Another alternative dosing strategy is based on two categories of BSA: for children with BSA 1.19 to 1.58 m^2^, 540 mg twice daily is recommended; for children with BSA > 1.58 m^2^, 720 mg twice daily is recommended [23]. However, there is no recommendation for children with BSA < 1.19 m^2^. Therefore, this study is aimed at developing a PPK model of MPA for pediatric patients treated with EC-MPS after renal transplantation with retrospectively collected data from the electronic medical records and routine therapeutic drug monitoring (TDM). With the model developed, initial dosing amount of EC-MPS was recommended for this population based on simulations.

## 2. Patients and Methods

### 2.1. Study Design and Data Collection

The protocol of this study complies with the ethical guidelines of the 1975 Declaration of Helsinki and was approved by the Institutional Review Board of Children's Hospital of Fudan University (No. (2020) 490). Written informed consent was waived because of the retrospective nature of this study. In this study, pediatric patients included were less than 18 years old, had received renal transplant for more than ten days, and had been taking oral EC-MPS (Mycophenolate Sodium Enteric-coated Tablets, Myfortic®, Novartis Pharma Stein AG). Of them, patients who were hospitalized in Department of Nephrology in Children's Hospital of Fudan University from June 2018 to August 2019 were included as the modeling group, and patients who were hospitalized from September 2019 to July 2020 were set as the validation group. Data on demographic characteristics, biochemical tests, blood routine results, MPA measurement, dosing regimen of EC-MPS, and coadministered medications were collected from patients' medical records. BSA was estimated with the Mosteller formula $\text{BSA }\left({\text{m}}^{2}\right)=\sqrt{\text{Weight }\left(\text{kg}\right)\times \text{Height}\left(\text{cm}\right)/3600}$ [24]. Estimated glomerular filtration rate (eGFR) was calculated using the Schwartz formula [25]. All the patients had been taking EC-MPS with unchanged dosing amount and frequency ≥ five days and had reached steady state before TDM was performed. We followed the methods of Wang et al. 2020 [26] for blood sampling and MPA concentration quantification. Briefly, the blood samples used for MPA measurement were drawn from patients at 30 min before EC-MPS administration and at 20 min, 1, and 3 h after administration. MPA concentrations were determined with the enzyme-multiplied immunoassay technique using the Viva-E System (Siemens Healthcare Diagnostics, Eschborn, Germany). The lower limit of quantification was 0.1 *μ*g/mL, with the calibration range being 0.1-15.0 *μ*g/mL. Data below the lower limit of quantification (BLOQ) were kept in the PPK analysis, referring to a previous study concluding that incorporating BLOQ concentrations into PPK modeling had superior performance over other established BLOQ methods in bias and precision [27].

### 2.2. PPK Modeling

A PPK model for renal transplant children was developed with nonlinear mixed-effect modeling methods using the Monolix software (2019R1, Lixoft ©). A one-compartment structural model with double extravascular absorption and first-order elimination was used to describe the PK process of MPA. The double absorption is composed of a first-order absorption (rate constant *k*_*a*1_, fraction *F*) with a lag time (*T*_lag1_) and a simultaneous zero-order absorption (duration *T*_k02_, fraction 1-*F*) with a lag time longer than the first delay. The dosing amount of EC-MPS was converted to the equivalent MPA amount by multiplying it by 0.936 according to a previous study of EC-MPS [8]. As bioavailability could not be quantified, estimated clearance (CL) and volume of distribution (*V*_*d*_) were actually the apparent CL and *V*_*d*_. *C*_MPA_ is the mycophenolic acid concentration in human plasma. The diagram of one-compartment structural model as shown in Figure 1.

PK parameters were assumed to follow a log-normal distribution, and model equations were logarithmically transformed. The equation for each PK parameters was ln (*P*_*i*_) = ln (*P*_pop_) + *η*_pi_, in which *P*_*i*_ is the individual estimate of the parameter, *P*_pop_ is the population estimate of the parameter, and 𝜂_pi_ is the interindividual variability of the parameter, which has a mean of 0 and a standard deviation (SD) of 𝜔. Residual error was described using $C_{\text{obs}}=C_{\text{pred}}+\sqrt{a^{2}+{\left(b\times C_{\text{pred}}\right)}^{2}}\times \varepsilon$. *C*_obs_ is the observed MPA concentration, *C*_pred_ is the predicted MPA concentration, *a* and *b* are both error model parameters, and 𝜀 is a normally distributed variable that has a mean of 0 and an SD of 1.

Continuous covariates were included into the model using a stepwise approach with the formula *P*_*i*_ = *P*_pop_ × (Cov_*i*_/mean (Cov))^*θ*cov^, in which *P*_*i*_ is the individual estimate of the PK parameter, *P*_pop_ is the population typical value, Cov*_i_* is the covariate value for *i*^th^ individual, and *θ*_cov_ is the fix-effect parameter. Categorical covariates were included into the model using the formula *P*_*i*_ = *P*_pop_ × e^Covi×*θ*cov^. In the forward selection process, instead of trying all covariate blindly, *P* values derived from Pearson's correlation test for continuous covariate and analysis of variance (ANOVA) for categorical covariate were used to select the covariate that could be first added to the model. Likelihood ratio test (LRT) was then used as the accepting or rejecting criterion with a threshold of 0.05. Similarly, in the backward elimination, *P* values from Pearson's correlation test and ANOVA were used to select the first covariate in the model that should be removed, and LRT was set as the criterion with a threshold of 0.05.

### 2.3. Model Evaluation

Models' goodness-of-fit was evaluated using scatter plots of observed versus predicted MPA concentrations, as well as scatter plots of normalized predication distribution error (NPDE) across different predicted concentrations and NPDE over time since the last dose. Visual predictive check (VPC) was employed to check the overlap between predicted and observed concentrations of MPA over time. External validation of the final model was conducted with a new set of data collected from September 2019 to July 2020. Goodness-of-fit plots were used to check if the final model could well predict the MPA concentrations in a different group of patients. Prediction error of the external validation was assessed using mean prediction error (MPE), mean absolute prediction error (MAPE), and root mean squared error (RMSE). Below are the formulas of the three indices.

(1) $$\begin{array}{c} \text{MPE}\%=\frac{1}{n}\overset{n}{\underset{i=1}{\sum }}\left[\frac{C_{\text{pred}}-C_{\text{obs}}\;}{C_{\text{obs}}}\right]\times 100\%,\\ \text{MAPE}\%=\frac{1}{n}\overset{n}{\underset{i=1}{\sum }}\left[\frac{\left|C_{\text{pred}}-C_{\text{obs}}\right|}{C_{\text{obs}}}\right]\times 100\%,\\ \text{RMSE}=\sqrt{\frac{1}{n}\overset{n}{\underset{i=1}{\sum }}{\left(C_{\text{pred}}-C_{\text{obs}}\right)}^{2}.} \end{array}$$

*C*_pred_ represents the individual predicted concentrations by the final model. *C*_obs_ is the observed concentration of the patients in the validation group.

### 2.4. Dosing Regimen Simulation

To recommend initial dosing regimen for the pediatric population, 1000 virtual patients were simulated to evaluate the efficacy and toxicity under different dosing regimens. The treatment target of MPA for renal transplant patient is AUC_0-12h_ between 30 and 60 mg·h/L according to previous studies [6, 7]. Derived targets for patients who take different amounts of EC-MPS in the morning and the evening or who take EC-MPS every 8 or 16 or 24 or 48 hours were 60–120 mg·h/L for AUC_0-24h_ and 120–240 mg·h/L for AUC_0-48h_. The efficacy threshold is 30 mg·h/L (AUC_0-12h_), 60 mg·h/L (AUC_0-24h_), and 120 mg·h/L (AUC_0-48h_). The toxicity threshold is 60 mg·h/L (AUC_0-12h_), 120 mg·h/L (AUC_0-24h_), and 240 mg·h/L (AUC_0-48h_).

Simulated dosing regimens included all the possible combinations of dosing amount (180 mg/dose, 360 mg/dose, 540 mg/dose, and 720 mg/dose) and dosing intervals (8 hours, 12 hours, 16 hours, 24 hours, and 48 hours). Another regimen was a different dosing amount in the morning and the evening (360/180 mg, 540/360 mg, 720/540 mg, every 12 hours [morning/evening]). Considering the MPA-EC which cannot be split into smaller doses, we only simulated dosing amount with the smallest increment as 180 mg. The percentage of patients whose AUCs were within the target range was calculated as the percentage of target attainment (PTA, efficacy without toxicity). The percentage of patients who had AUCs above the efficacy threshold was denoted as the percentage of efficacy. The percentage of patients who had AUCs above the toxicity threshold was denoted as the percentage of toxicity.

## 3. Results

### 3.1. Patients

This study included 128 pediatric patients, among which 96 were in the modeling group and 32 were in the validation group. The modeling group consisted of 52 boys and 44 girls, with a median age of 13.3 (range 4.3–18.0) years, a median height of 147 (102–171) cm, a median weight of 39.0 (15.0–67.0) kg, and a median BSA of 1.26 (0.66–1.78) m^2^. 94 out of the 96 patients took tacrolimus concomitantly, and the other 2 patients coadministered cyclosporin. The validation group consisted of 15 boys and 17 girls, at a median age of 13.0 (3.6–18.3) years, a median height of 148 (104-171) cm, a median weight of 36.5 (12.7–74.0) kg, and a median BSA of 1.22 (0.61–1.80) m^2^. The demographic, clinical, biological, and pharmacological data of the modeling and validation groups are listed in Table 1.

### 3.2. PPK Model

A one-compartment structural model with double extravascular absorption and first-order elimination was developed. BSA was added as a covariate of the clearance to the final model with -2× log-likelihood decreasing from 1352 to 1339. The final model equations are *k*_a1i_ (1/*h*) = *θ*_ka1_, *T*_k02_ (*h*) = *θ*_Tk02_, *F* = *θ*_*F*_, *T*_lag1i_ (*h*) = *θ*_Tlag1_, diffT_lag2_ (*h*) = *θ*_diffTlag2_, *V*_*i*_ (*L*) = *θ*_*V*_, and CL_*i*_ (*L*/*h*) = *θ*_CL_ × (BSA/1.23)^*θ*_CL-BSA_^, where *θ*_ka1_, *θ*_Tk02_, *θ_F_*, *θ*_Tlag1_, *θ*_diffTlag2_, *θ_V_*, *θ*_CL_, and *θ*_CL-BSA_ were estimated to be 0.123, 2.90, 0.553, 8.45, 5.78, 3.73, 4.28, and 1.30, respectively. The parameters estimated from the base model and the final model are presented in Table 2. The goodness-of-fit of the final model is presented in Figure 2. The scatter plots of observed versus predicted concentrations are presented in the logarithmic scale. The points in the scatter plot of observed concentrations versus individual predicted concentrations are well distributed along the line of *y* = *x*. The VPC plot is shown in Figure 3. The 10^th^, 50^th^, and 90^th^ percentiles of the observed data fall well within the 95% confidence interval of the predicted 10^th^, 50^th^, and 90^th^ percentiles, except for an outlier in the 10^th^ percentile. The result of the external validation of the final model with another set of data is presented as a scatter plot of observed versus individual predicted concentrations in Figure 4. The prediction errors of the external validation are shown in Table 3. The RMSE is 0.810 mg/L, and the MAPE is 10.0%.

### 3.3. Dosing Regimen Simulation

The results of simulation are depicted in Figures 5–7. 1000 pediatric patients with uniformly distributed BSA from 0.22 m^2^ to 2.03 m^2^ are simulated. The virtual patients are divided into 6 groups with different ranges of BSA. The range of BSA was referred to 2000 CDC Growth Charts [28]. The highest PTA among all the groups and all the dosing regimens are around 50%, meaning most pediatric patients have either overly high exposure to MPA or overly low exposure to MPA when treating with EC-MPS. For patients with BSA of 0.22–0.46 m^2^, the best dosing regimen is 180 mg every 48 hours. For patients with BSA of 0.47–0.67 m^2^, the best dosing regimen is 180 mg every 24 hours. For patients with BSA of 0.68–0.96 m^2^, the best dosing regimen is 180 mg every 24 hours. For patients with BSA of 0.97–1.18 m^2^, the best doing regimen is 360 mg every 24 hours. For patients with BSA of 1.19–1.58 m^2^, the best doing regimen is 540 mg every 24 hours. For patients with BSA of 1.59–2.03 m^2^, the best dosing regimen is 360 mg every 12 hours.

## 4. Discussion

This study is the first to develop a PPK model of EC-MPS in the pediatric population. From the model parameter estimates, we can tell that there is a significant delay in absorption after oral administration of EC-MPS. The first absorption lag time is 8.45 hours, and the second absorption lag time is 5.78 hours longer than the first absorption. About 55.3% of the EC-MPS is absorbed through first-order absorption pathway at an earlier time, and the rest is absorbed through zero-order absorption pathway at a later time. The apparent volume of distribution of MPA is about 3.73 L. The typical value of apparent clearance for a pediatric patient with BSA of 1.23 m^2^ is about 4.28 L/h.

There is a previous study in the adult renal transplant population by de Winter et al. that compared the PPK characteristics of EC-MPS and MMF [8]. It developed a two-compartment model with a lag time in absorption to describe the PK process of both EC-MPS and MMF. The results showed that EC-MPS had longer lag time in absorption than MMF, and the *T*_lag_ was more variable following the administration of EC-MPS, varying between 0.9 h and 5.5 h with a median of 2.0 h for morning dose and between 5.4 h and 12.3 h with a median of 8.9 h for evening dose. The absorption lag time in our study is longer than the morning lag time in de Winter et al.' study and is close to the lag time of evening administration of EC-MPS in their study. Since all the blood samples in our study were collected in the morning, we did not develop separate models for morning PK and evening PK. The long lag time in absorption of EC-MPS could be due to both the enteric-coated feature of this particular formula and the EHC characteristic of MPA. The discrepancy between morning absorption and evening absorption could be explained by the differences in gastrointestinal movement rate and environment of the two time periods [29]. Further research is warranted by collecting blood samples after evening administration of EC-MPS to gain better insights into the variations of absorption in different time of the day.

Most of the patients in our study used tacrolimus concomitantly, and only two patients in the modeling group coadministered cyclosporin. It was reported that cyclosporin inhibits the MPAG transporting from hepatocytes into the bile, thus decreasing the EHC [30]. On the contrary, tacrolimus does not significantly affect the PK of MPA, as was showed in a study by van Gelder et al. [31]. Another study in transplant children compared the effects of cyclosporin and tacrolimus, the result of which showed that coadministered cyclosporin instead of tacrolimus increased the clearance of MPA by 63% [6]. The clearance of MPA estimated for the children on tacrolimus in the study above is 5.51 L/h, which is close to the clearance estimated to be 4.28 L/h in our study.

BSA was added as a covariate for clearance, which improved the model fitting. With the increase in BSA, the clearance of MPA increases, which is in accordance with previous PPK studies adding weight as a covariate to the model of MPA [6, 22]. Current dosing guidance from the “Pediatric & Neonatal Dosage Handbook” for EC-MPS usage on renal transplant children is also based on the BSA [23]. For children aged 5 years or older, 400 mg/m^2^/dose twice daily is recommended on the book. Since the enteric-coated tablet of MPS should not be split so as not to dissolve until reaching the intestine, the alternative recommendation might be more practical, which suggested 540 mg twice daily for children with BSA of 1.19–1.58 m^2^ and 720 mg twice daily for children with BSA over 1.58 m^2^. Considering the MPS amount per tablet is 180 mg, we only simulated dosing regimens of different dosing frequencies combined with different dosing amounts that are divisible by 180. The simulation results showed that the overall target range attainment rate for all the children with different BSA is quite low under different dosing regimens of EC-MPS, with the highest percentage around 50%. For children with BSA lower than 0.67 m^2^, the twice daily dosing frequency could be too much to safely achieve the immunosuppressive target range. For children with higher BSA, 180 mg per tablet could not help reach precision treatment since it cannot be split into smaller increment. Therefore, small enteric-coated pellets with lower MPS amount per unit are worth developing to attain both goals of prescribing more precisely in the pediatric population and minimizing the gastrointestinal adverse reactions caused by the drug.

Previous studies have reported that MPA predose trough concentration (*C*_0_) correlates poorly with AUC [8, 32]. In our study, the correlation coefficient between the AUC and *C*_0_ is 0.304, which is consistent with the previously reported. To improve the accuracy of TDM, AUC is often used in replacement of trough concentration to measure the exposure of MPA. MPA-AUC_0-12h_ of 30 to 60 mg·h/L is generally recognized as the treatment target. Kiberd et al. [33] found that AUC_0−12h_ < 30 mg · h/L would identify 79% of patients with rejection within first 3 months posttransplantation. Although better efficacy can be achieved by increasing the dosing amount, toxicity of the drug should not be overlooked. Potential adverse reactions of MPA include leucopenia, infections, and diarrhea [11, 30, 34]. The cut-off value of AUC_0-12h_ for toxicity was suggested as 60 mg·h/L [11, 16]. However, there is no definitive upper range for toxicity since there were many issues regarding the design of the studies that assessed the toxicity of MPA [7, 11]. Risks and benefits associated with the exposure targets of MPA should be weighed carefully for each patient before making individualized treatment plan. In the first few months after transplantation, the adverse consequences of rejection are usually greater than the negative effect brought by the toxicity of MPA; so, the exposure target could be set as high as 70 mg·h/L for patients at much higher risk of rejection [11].

## 5. Conclusions

A PPK model of EC-MPS has been developed in renal-transplant pediatric patients. Clearance of MPA was varied with the BSA. Optimal initial dosing regimens are recommended based on BSA. For patients with BSA of 0.22–0.46 m^2^, the best dosing regimen is 180 mg every 48 hours. For patients with BSA of 0.47–0.67 m^2^, the best dosing regimen is 180 mg every 24 hours. For patients with BSA of 0.68–0.96 m^2^, the best dosing regimen is 180 mg every 24 hours. For patients with BSA of 0.97–1.18 m^2^, the best doing regimen is 360 mg every 24 hours. For patients with BSA of 1.19–1.58 m^2^, the best doing regimen is 540 mg every 24 hours. For patients with BSA of 1.59–2.03 m^2^, the best dosing regimen is 360 mg every 12 hours. Considering the inflexibility of the current dosage form of MPS, future development of smaller amount per tablet suitable for younger children is warranted.

## Figures and Tables

**Figure 1:** Diagram of one-compartment structural model.

**Figure 2:** Goodness-of-fit plots for the final model of mycophenolic acid. (a) Observed versus population predicted concentrations in logarithmic scale. (b) Observed versus individual predicted concentrations in the logarithmic scale. (c) Normalized prediction distribution error (NPDE) across predicted concentrations. (d) NPDE over time since last dose.

**Figure 3:** Visual predictive check of concentrations over time since last dose. The blue lines represent the 10^th^, 50^th^, and 90^th^ percentiles of observed data, and the three areas represent the 95% confidence interval of the predicted 10^th^, 50^th^, and 90^th^ percentiles. MPA: mycophenolic acid.

**Figure 4:** Observed versus individual predicted concentrations of external validation of the final model with a new set of data.

**Figure 5:** Percentage of efficacy under different dosing regimens of enteric-coated mycophenolate sodium from simulation. Different colored lines represent patients with different body surface areas (BSA). The efficacy threshold of area under the concentration-time curve (AUC) of mycophenolic acid is 30 mg·h/L (over 12 hours after last dose, AUC_0-12h_), 60 mg·h/L (over 24 hours after last dose, AUC_0-24h_), and 120 mg·h/L (over 48 hours after last dose, AUC_0-48h_). (a) One dose every 8 hours (q8h). (b) One dose every 12 hours (q12h). (c) One dose every 16 hours. (d) One dose every 24 hours (qd). (e) One dose every 48 hours (qod). (f) One dose every 12 hours (different dosing amounts in the morning and the evening).

**Figure 6:** Percentage of toxicity under different dosing regimens of enteric-coated mycophenolate sodium from simulation. Different colored lines represent patients with different body surface areas (BSA). The toxicity threshold of area under the concentration-time curve (AUC) of mycophenolic acid is 60 mg·h/L (over 12 hours after last dose, AUC_0-12h_), 120 mg·h/L (over 24 hours after last dose, AUC_0-24h_), and 240 mg·h/L (over 48 hours after last dose, AUC_0-48h_). (a) One dose every 8 hours (q8h). (b) One dose every 12 hours (q12h). (c) One dose every 16 hours. (d) One dose every 24 hours (qd). (e) One dose every 48 hours (qod). (f) One dose every 12 hours (different dosing amounts in the morning and the evening).

**Figure 7:** Percentage of target range attainment (PTA) under different dosing regimens of enteric-coated mycophenolate sodium from simulation. Different colored lines represent patients with different body surface areas (BSA). The target range of area under the concentration-time curve (AUC) of mycophenolic acid is 30-60 mg·h/L (over 12 hours after last dose, AUC_0-12h_), 60-120 mg·h/L (over 24 hours after last dose, AUC_0-24h_), and 120-240 mg·h/L (over 48 hours after last dose, AUC_0-48h_). (a) One dose every 8 hours (q8h). (b) One dose every 12 hours (q12h). (c) One dose every 16 hours. (d) One dose every 24 hours (qd). (e) One dose every 48 hours (qod). (f) One dose every 12 hours (different dosing amounts in the morning and the evening).

**Table 1:** Demographic, clinical, biochemical, and medication usage data of modeling and validation groups.

Variable	Group for modeling	Group for validation	*P* values^∗^
Sex (M/F)	96 (52/44)	32 (15/17)	1
Age (years)	13.3 (4.3–18.0)	13.0 (3.6–18.3)	0.802
Height (cm)	147 (102–171)	148 (104–171)	0.908
Weight (kg)	39.0 (15.0–67.0)	36.5 (12.7–74.0)	0.486
BSA (m^2^)	1.26 (0.66–1.78)	1.22 (0.61–1.80)	0.577
Posttransplant days (days)	396 (13–2258)	600 (19–2158)	0.184
SCR (*μ*mol/L)	65.0 (35.0–272.0)	63.0 (42.0–150.0)	0.754
CLCR (mL/min/1.73 m^2^)	78.8 (20.1–164.6)	75.6 (37.7–126.4)	0.809
BUN (mmol/L)	7.30 (3.10–28.50)	6.10 (3.30–12.40)	0.200
ALT (IU/L)	12.1 (4.5–140.3)	13.5 (6.5–68.2)	0.488
AST (IU/L)	22.0 (12.0–60.2)	22.7 (13.8–199.3)	0.338
DBIL (*μ*mol/L)	2.70 (0.90–5.10)	2.75 (1.20–8.60)	0.657
TBIL (*μ*mol/L)	7.60 (3.00–20.00)	6.60 (2.50–11.60)	0.046
ALB (g/L)	41.4 (31.0–49.8)	41.4 (36.6–54.9)	0.229
GLB (g/L)	28.1 (17.1–46.6)	26.6 (19.0–39.4)	0.122
TCH (mmol/L)	4.09 (2.30–7.20)	3.56 (2.73–5.55)	0.021
LDH (IU/L)	243 (141–485)	250 (166-2193)	0.509
PLT (×10^9^/L)	240 (101-451)	259 (139-385)	0.690
WBC (×10^9^/L)	6.65 (2.50–19.60)	6.00 (2.00–14.30)	0.364
RBC (×10^12^/L)	4.43 (2.18–7.36)	4.37 (2.83–6.87)	0.888
HGB (g/L)	116 (72–167)	119 (87–151)	0.974
Total number of samples	384	125	
Dosing amount (mg/kg/day)	10.5 (3.4–24.0)	10.6 (3.7–19.8)	0.389
Dosing amount (mg/m^2^/day)	325 (117–605)	305 (124-514)	0.217
Comedications			
Tacrolimus	94 (97.9%)	32 (100%)	0.429
Cyclosporin	2 (2.08%)	0 (0%)	1

Data are presented as *n* (percentage) or median (range). BSA: body surface area; SCR: serum creatinine; CLCR: creatinine clearance; BUN: blood urea nitrogen; ALT: alanine aminotransferase; AST: aspartate aminotransferase; DBIL: direct bilirubin; TBIL: total bilirubin; ALB: albumin; GLB: globulin; TCH: total cholesterol; LDH: lactate dehydrogenase; PLT: platelet; WBC: white blood cell; RBC: red blood cell; HGB: hemoglobin; IVIG: intravenous immune globulin. ^∗^For continuous variables, Mann–Whitney test was used to compare the difference between the two groups. For categorical variables, chi square test was used.

**Table 2:** Parameter estimates from the base model and final model.

Parameters	Base model		Final model	
	Estimate	RSE/%	Estimate	RSE/%
Structure model parameters				
𝜃_ka1_	0.112	21.4	0.123	20.5
𝜃_Tk02_	1.03	69.7	2.90	42.1
𝜃*_F_*	0.644	6.12	0.553	6.30
𝜃_*T*lag1_	8.40	7.71	8.45	9.30
𝜃_diff*T*lag2_	5.76	16.5	5.78	18.0
𝜃*_V_*	4.63	22.6	3.73	13.0
𝜃_CL_	4.29	7.43	4.28	6.53
𝜃_CL-BSA_	\	\	1.30	20.4
Interindividual variability				
𝜔_ka1_	1.14	15.7	0.885	15.2
𝜔_Tk02_	3.34	40.5	2.31	19.1
𝜔_F1_	0.747	18.4	0.513	18.8
𝜔_*T*lag1_	0.478	11.4	0.576	11.3
𝜔_diff*T*lag2_	0.688	24.7	0.941	33.6
𝜔*_V_*	0.840	18.3	0.337	26.3
𝜔_CL_	0.504	10.1	0.481	13.3
Residual error model parameters				
*a*	0.0709	41.4	0.0631	25.2
*b*	0.199	7.57	0.199	7.5

This PK model has a double extravascular absorption composed of a first-order absorption (rate constant *k*_a1_, fraction *F*) with a lag time (*T*_lag1_) and a simultaneous zero-order absorption (duration *T*_k02_, fraction 1-*F*) with a lag time longer than the first delay (*T*_lag2_ = *T*_lag1_ + diff*T*_lag2_). The PK model has a central compartment (volume *V*) and a linear elimination (clearance CL). The final model included body surface area (BSA) as the covariate for CL. Final model equations: *k*_a1i_ (1/*h*) = *θ*_ka1_, *T*_k02_ (*h*) = *θ*_Tk02_, *F* = *θ*_*F*_, *T*_lag1i_ (*h*) = *θ*_*T*lag1_, diff*T*_lag2_ (*h*) = *θ*_diff*T*lag2_, *V*_*i*_ (*L*) = *θ*_*V*_, CL_*i*_ (*L*/*h*) = *θ*_CL_ × (BSA/1.23)^*θ*_CL-BSA_^. 𝜃_ka1_, 𝜃_Tk0_, 𝜃*_F_*, 𝜃_*T*lag1_, 𝜃_diffTlag2_, 𝜃*_V_*, and 𝜃_CL_ are typical values of *k*a1, *T*k02, *F*, *T*lag1, diffTlag2, *V*, and CL, respectively; 𝜃_CL-BSA_ is the typical value of the power of the covariate BSA for the CL. 𝜔_ka1_, 𝜔_Tk02_, 𝜔_F1_, 𝜔_Tlag1_, 𝜔_diffTlag2_, 𝜔*_V_*, and 𝜔_CL_ are standard deviations of interindividual random effects of the ka1, Tk02, *F*, Tlag1, diffTlag2, *V*, and CL, respectively. *a* and *b* are residual error model parameters from the equation *C*_obs_ = *C*_pred_ + sqrt [*a*^2^ + (*b* × *C*_pred_)^2^] × *ε*; sqrt: square root; 𝜀 is a normally distributed variable that has a mean of 0 and a standard deviation of 1. RSE: relative standard error.

**Table 3:** Prediction error of external validation.

Indices	Value
MPE (%)	-0.880
MAPE (%)	10.0
RMSE (mg/L)	0.810

MPE: mean prediction error; MAPE: mean absolute prediction error; RMSE: root mean squared error.

## Data Availability

All the original data for this study can be accessed by contacting the corresponding author upon reasonable request.
